The article "Environmental Emission Validation Analysis Using a Dual-Fuel Engine" was published in 2022. Journal: J Environ Public Health.

# Environmental Emission Validation Analysis Using a Dual-Fuel Engine

**DOI:** 10.1155/2022/9852220

**Published:** 2022-08-25

**Authors:** Karthikeyan S, Arif Senol Sener, Bothichandar T

**Affiliations:** ^1^Department of Mechanical Engineering, Syed Ammal Engineering College, Landai, Tamilnadu, India; ^2^Department of Mechanical Engineering, Engineering and Architecture Faculty, Nisantasi University, Istanbul, Turkey; ^3^Faculty in Industrial Engineering Department, SMIE, Ambo University, Ambo, Ethiopia

## Abstract

The research work presents the results of testing using an internal combustion engine ignition/compression using diesel and LPG mixtures without preheating. The energy performance of regulated brake emissions and changes in fuel consumption for a compression ignition engine is investigated in this study. It is assured that the engine's operation is not harmed as a result of the installation of this mix. The engine produces torque and power when it is working according to the design parameters. In tests with these combinations, results with a thermal efficiency of 10% were obtained, which was higher than the 5% obtained in diesel tests. It is used in compression ignition engines to offer a fuel source for the generation of electrical energy.

## 1. Introduction

Currently, about 60% of the oil produced in the world is used to produce fuel for fuel system transportation. The greatest challenges that the world has are access to energy, environmental sustainability, security, and development for economic growth [1]. Therefore, it is given as a solution to liquefied petroleum gas (LPG). LPG is a fuel derived from the mixture of propane and butane. The first is present in large quantities, and the second may be in low percentages; these are obtained from natural gas deposits or distillation petroleum [2]. This project aims to check whether the diesel-LPG mixture without preheating and without substantial modifications to the internal combustion engine of compression ignition can operate adequately, and to further study whether the engine is properly operated, then the behavior of emissions such as carbon dioxide (CO_2_), carbon monoxide (CO), and unburned hydrocarbons (HC). On the contrary, the economic benefits are due to the difference in fuel prices, especially when assessing diesel fuel with different volumetric flow rates compared with when assessing LPG. Internal combustion engines are part of the most energy generators currently used, and their main function is to change the chemical energy produced by mechanical energy fuel [3]. Due to their great versatility, they are used in various applications such as land and sea transportation, plant power generators, and non-interconnected areas, that is, places where the possibility of having energy is minimal. The generation of electricity using an internal combustion engine is a solution to the lack of energy. This is one of the most used motors in the industry, such as compression/ignition. One of the disadvantages of compression/ignition engines is the emissions generated when operating [4].

For this reason, it is desired to make a mixture of diesel and LPG to study the effects that combustion of these can have on emissions and therefore know whether there is a reduction in consumption of the fuel by the addition of LPG. On the contrary, it is important to expand knowledge about diesel-LPG (dual-fuel) engines to contribute to an energy solution at the national level [5]. With the implementation of diesel-LPG mixture as a fuel in a combustion engine internally, a considerable decrease is expected in the particles expelled in the exhaust gases, promoting care for the environment, in addition to benefiting sectors that lack electricity service [6]. LPG is a natural hydrocarbon fuel consisting of propane and butane in any percentage. When pressure is applied, it liquefies, allowing storage of a large quantity versus a small volume. Many cars worldwide use this gas since it has low cost, is environmentally friendly, generates better performance, and is safe to use [7]. A better combustion rate of LPG than that of diesel helps extend the engine's life; it is also a noncorrosive, additive-free gas with an octane good rating. The addition of LPG before the turbocharger reduces the air temperature, thus favoring the air-gas mixture that later burns with diesel, which is used as an additional fuel instead of a substitute fuel. A study of liquefied petroleum gas as an alternative motor fuel shows how to combine diesel with LPG to reduce polluting gas emissions [8]. They created an injection system for the gas, which is remotely controlled using a computer injected according to the engine requirement; it was concluded that when revolutions increase by a minute of the engine, the CO decreases and NOX increases. In another instance, the use of liquefied petroleum gas has more advantages than disadvantages [9]. However, its most notable flaw is the stored way it is made in pressure tanks and is later distributed. Safety is an important factor, and the transport of LPG can threaten it. For example, there have been several accidents where LPG explodes; however, they have been minimized with the rules that have been stipulated [10]. Another interesting aspect is the great expectation of implementing the LPG as an alternative fuel within the automotive industry and even transitioning to other more environmentally friendly energy sources. Regarding the design and regulations for converting motor vehicles with gasoline to those with LPG, many books and other literature discuss the performance and LPG engine efficiency through experiments, models, and simulations [11]. Finally, the following work combines two fuels, diesel and liquefied petroleum gas, which is developed to guarantee that a combination of fuels can reduce the polluting gases generated by diesel and observe their behavior in terms of efficiency, and delivered torque and power.

The main contribution of a dual-fuel engine application is to provide a lower compression pressure and a longer ignition delay than a diesel engine in the normal mode. A dual-fuel engine has a higher output power than a single-fuel engine. Although dual-fuel engines emit significantly less carbon monoxide (CO), carbon dioxide (CO2), and hydrocarbons (HC) than single-fuel engines, the exhaust gases emitted by dual-fuel engines are significantly cleaner.

Dual-fuel engines have specific gaps in specific areas in order to achieve the highest substitution ratio or the highest percentage of natural gas replaced by diesel fuel. A small amount of diesel can be accurately and consistently injected into an engine, which currently limits this ratio.

## 2. Experimental Setup

Modifications were made before starting the experimental tests, such as assembling a flow valve at the diesel inlet to the engine to have greater control of the fuel flow, as shown in Figure 1. Moreover, to measure the temperature in the oil, the exhaust pipe, and the pipe air intake, three thermocouples were introduced. During the first tests, while evaluating the correct operation of the test bench, the universal coupling showed stud/thread faults that hold the wedge, increasing the play of the part and affecting the measurements of the torque sensor consequently [12]. The thread diameter was changed with the help of a male and fitted with a prisoner. The installation of the independent fuel tank is carried out for the intake of the fuel at the same time since the last tank located at a side of the engine made it difficult to take data with the digital camera.  Table 1 shows the uncertainty error using the test engine.

## 3. Experimental Procedure

Then, the start button is pressed, and automatically, the program says calibration in progress. When the calibration screen disappears, the program begins to collect data [13]. The probe should therefore be placed on the exhaust pipe and monitored until the values of the exhaust gas leakage stabilize [14]. It is recommended to clean the probe or cable of the gas analyzer with the help of a compressor after each intake so that the next data can be taken. In another instance, with the help of a digital hygrometer thermometer, the ambient temperature and relative humidity data values are taken last after having the data of the gases of the exhaust gas analyzer. At the end of the data records for the loads mentioned above, it is necessary to remove the load and turn off the engine to let it cool down and thus start the procedure again. After about 5 minutes, the above procedure mentioned for each diesel-LPG mixture is repeated. However, this time the flow of the LPG supplied has to be taken into account [15]. This flow is controlled by a flow meter, which measures the volumetric flow rate in standard cubic feet per hour (SCFH). Before braking the engine with various loads, the liquid petroleum gas shut-off valve is opened, and the corresponding data are collected for each load.  Table 2 shows the three flows used in practice and their real values. Corresponding to the volumetric flow (gr/s), Table 2 also shows the uncertainty error using the test engine.

## 4. Results and Discussion

Next, the results were obtained with the four types of fuels in their mixture, evidencing the behavior of each of these to the same loads, following the same procedure and trying that this is a cause of change in the conditions of the tests.

### 4.1. Specific Fuel Consumption

The specific brake fuel consumption results for each test are shown in Figure 2. The diesel-LPG 1 mixture has 12% more consumption at low loads than diesel, but when working with loads, it is better to use the diesel-LPG 1 mixture with a saving of 63% of fuel. The specific fuel consumption fuel in the diesel-LPG 2 mixtures saves 30% and in the diesel-LPG mixtures saves 3.45% of fuel, being a favorable option to reduce consumption in loads whether it can be low or high [16].

### 4.2. Thermal Efficiency

Consequently, in Figure 3, it can be seen that the thermal efficiency depends on the amount of fuel that enters the cylinder [17]. The less the diesel is incorporated into the cylinder, the engine will take better advantage of the heat produced by the combustion of the mixtures. This is evidenced by the specific fuel consumption in Figure 2, knowing that the volume of air inside the cylinder can only be affected by the ambient temperature when the tests were done, and that the amount of fuel makes the difference that the mixture can be rich or poor in the air since the air inside the motor is constant [18]. This means that the less the fuel entered into the cylinder, the air-fuel ratio will be better regarding diesel. On the one hand, for the higher load applied to diesel, there is a decrease in the thermal efficiency of 64%; on the other hand, the mixtures of diesel-LPG 1, diesel-LPG 2, and diesel-LPG 3 presented a reduction in the thermal efficiency of 47%, 74%, and 76%, respectively.

### 4.3. Volumetric Efficiency

The average values of the ambient temperature and the relative humidity with which each test was carried out were recorded [19]. The temperature directly influences the volumetric efficiency of the engine; it decreases the density of air. From Figure 4, it can be inferred that the lower the temperature, the higher the humidity and therefore the higher the volumetric efficiency for the mixtures than for diesel as there is an increase in air volume.

### 4.4. Carbon Dioxide Emissions

Carbon dioxide emissions in Figure 5 show a decreasing trend. This implies that as the load increases, the motor has a lean air-fuel ratio in air [20]. This occurs because of the amount of fuel that is injected into the cylinder when the butterfly valve opens. A reduction in CO_2_ percentage was only observed for GLP 1, GLP 2, and GLP 3 mixtures when 80% of the load was applied. The combustion process is not complete by varying only 5% volumetric efficiency. The result of this is that there is insufficient oxygen to react with CO_2_ in the atmosphere.

### 4.5. Carbon Monoxide Emissions

Carbon monoxide emissions are linked to carbon dioxide emissions. Carbon is inversely proportional to the air-fuel mixture since when combustion occurs inside the cylinder if and only if there is a lean air-fuel mixture, the reaction generates carbon monoxide as a consequence of the lack of oxygen to react to carbon dioxide. In Figure 6, the diesel produced higher CO emissions for all applied loads than mixtures [21–23]. It can be seen that emissions in all cases tend to increase when the load is greater.

### 4.6. Unburned Hydrocarbon Emissions

The use of mixtures at low loads is not suitable due to the generation of unburned hydrocarbons, being increased by 74% up to 16.4% (Figure 7). In order to achieve low emissions of HC with respect to diesel fuel, it is necessary to make the engine work with high loads, that is, in a range of 80% to 100% [24].

### 4.7. Operating Cost per Hour of the Engine

According to Figure 8, diesel fuel consumption decreases when mixed with GLP; these values are positive for research since it complies with one of the specific objectives. The cost for diesel-LPG mixture 1 drops by only 3%, which is smaller, when a 20% load is applied. However, it has a decrease of 65% for the applied load of 100%. On the contrary, the diesel-LPG 2 mixture reduces the cost of low-load fuel by 28% and the high-load (100%) fuel by 47%. Finally, the diesel-LPG mixture 3 reduced costs by 29% for low loads and 74% for higher loads [25]. It should be noted that these percentages come out of the relationship between diesel as a reference and the costs of mixtures recorded [9].

## 5. Conclusions

The use of diesel-LPG mixtures without preheating below 80% of the load is not recommended because the combustion ratio inside the cylinder is poor in air, which does not allow this mixture to be used generating up to 16.3% of HC emissions, which are higher than those of diesel as opposed to when the engine works with loads in a range of 80% to 100%, which allows these emissions drop from 18% to 97% depending on the load. If it is necessary to reduce diesel consumption, it is recommended to increase the percentage of LPG in the fuel mixture since compared with the diesel-LPG mixture 2 and diesel-LPG 3 without preheating, the specific fuel consumption had a 20% decrease, which can generate an economic saving for power generation. The decrease in CO emissions and the increase in CO_2_ confirm that the diesel-LPG blends without preheating have a rich air-fuel ratio with a minimum of 13% and a maximum of 17.9% and that diesel allows the oxygen obtained from the air to react adequately with CO to produce CO_2_. The increase in thermal efficiency from 6% to 28.5% when working with the diesel-LPG mixture without preheating compared with when working with diesel is a positive indicator of engine performance, confirming that this mixture is effective for ignition engine compression and a possible alternative fuel for generating electrical energy. Compared to diesel-LPG blends without preheating, the best results were obtained with diesel-LPG 3, since it has a minimum thermal efficiency of 28%, a maximum thermal efficiency of 28.5%, and a reduction in diesel consumption on average of 45%. However, one of the factors to consider for this mixture is the load with which it works optimally since loads are less than 40%; the engine did not stabilize due to the lack of mass of the air and the low revolutions per minute. In comparison with previous studies, the LPG energy substitution can be accomplished up to 50% at lower loads and up to 25% at higher loads. Pure diesel engines perform better than a mixture of diesel and gasoline up to about 50% of loading on the engine. There are numerous advantages of operating the engine in a dual-fuel mode over operating it in a pure diesel mode at higher engine loads.

## Figures and Tables

**Figure 1:** Schematic diagram of the proposed diesel-LPG (dual-fuel) system.

**Figure 2:** Brake-specific fuel consumption vs load.

**Figure 3:** Thermal efficiency vs load.

**Figure 4:** Volumetric efficiency vs load.

**Figure 5:** Carbon dioxide vs load.

**Figure 6:** Carbon monoxide vs load.

**Figure 7:** Hydrocarbon vs load.

**Figure 8:** Cost analysis vs load.

**Table 1:** Uncertainty error using the test engine.

Parameter	Resolution	Accuracy	Range
CO	1 ppm	±20 ppm (for <400 ppm CO)	0–10000 ppm
HC	0.3%	±10 ppm (for <100 ppm HC)	0–5000 ppm
Oxygen (O_2_)	0.1%	−0.1% + 0.2%	0–25%
Carbon dioxide (CO_2_)	0.1%	±0.3%	0–fuel value
Pressure	0.01 mbar	±0.5% full scale	0–150 mbar
Operating temperature, −10 to 45°C			
Warm-up time, 3 min			
Response time T90, 30 sec			
Operating humidity, 5–95% noncondensing			

**Table 2:** LPG flow for the three different tests.

Designation	Flow (SCFH)	ṁ LPG (gr/s)
Diesel-LPG 1	5	4.80 E-08
Diesel-LPG 2	10	9.70 E-08
Diesel-LPG 3	15	1.40 E-07

## Data Availability

The data used to support the findings of this study are included in the article.
